# Research on Fitness Movement Monitoring System Based on Internet of Things

**DOI:** 10.1155/2022/5120556

**Published:** 2022-03-08

**Authors:** Zhenhao Yu

**Affiliations:** Shanxi University, Taiyuan 030006, China

## Abstract

A multiuser motion-monitoring system based on MEMS is proposed for fitness movement, it is used to monitor the three important parameters of movement type, movement times, and movement cycle in the body movement and supports the simultaneous use of multiple users. The specific content of the method: (1) In terms of system design, a motion-monitoring system framework based on the Internet of things is proposed considering the motion-monitoring scene oriented to intelligent fitness. (2) In the aspect of algorithm, the relevant research of motion pattern recognition and cycle calculation method is carried out. For action pattern recognition, SVM-based algorithm to adapt to different computing capabilities of the scene is applied. (3) Experiments on 7 kinds of actions show that the proposed deep neural network has a good learning effect on small datasets, the recognition accuracy of the proposed deep neural network reaches 97.61%, and the recognition accuracy of SVM also reaches over 96%. In the 50 times of operation cycle calculation experiments, the frequency statistics algorithm has reached 100% of the calculation accuracy, and the calculation results of the operation cycle are close to the real value, which proves the validity of the method of cycle calculation. The experiment proves that the zero-crossing detection and wavelet analysis methods have a good overall effect and can accurately count and calculate the period when the number of actions is more, improve fitness efficiency, and provide guarantee for human health.

## 1. Introduction

In today's society, the times are constantly developing, and people's requirements for material life will gradually improve, living standard has been satisfied at the same time, began to pursue a healthy lifestyle, and basically is based on physical exercise. Running is one of the most important activities for people to carry out physical exercise, it is one of the most popular fitness activities in the world at present, it is highly evaluated in the medical and sports circles, and it is also the most scientific and effective way to keep one's body and mind. It can effectively strengthen the muscle and bone function of the limbs, improve the cardiopulmonary function, and play a great role in weight loss [1]. At present, more popular sports exercise tools or fitness equipment have been developed. With the development of society, some jobs require people to have a good physical fitness to adapt, which strengthens the importance of physical exercise, but due to the restriction of some objective factors, such as climate, environment, and venue, people pay more and more attention to indoor exercise, and treadmill fitness has become the preferred way for people to exercise [2]. From a physical point of view, on the ground or on a treadmill, the motion is almost the same, but from a mechanical point of view, on a treadmill, since the belt can drive the lower limbs, the movement force and force become more flexible, which can save people's leg force [3]. It is conceivable that the treadmill enters the gym or home as a matter of course [4]. In the process of physical exercise, guidance from professionals is essential. Nowadays, in most places for physical exercise, such as gyms, rehabilitation training centers and physical education classes in schools, there are coaches or related professionals to demonstrate the correct movements and monitor the movement status of the athletes. No matter in the field of fitness, rehabilitation training or physical education, correct exercise under the guidance of professionals is an important guarantee to improve the training effect and prevent sports injury. At present, the portable equipment or large medical equipment used for monitoring the basic parameters of the human body has little value except for recording and monitoring [5]. From the point of view of the bodybuilder, it is not to bring the best fitness effect. In view of the above situation, the combination of treadmill fitness and sports health monitoring, the collection and storage of fitness people in the running of the physiological parameters, and through certain analysis and processing, the body and sports conditions of the bodybuilders are presented in time, so that the bodybuilders can check their current health index in real time and understand their exercise situation [6]. Therefore, the domestic and foreign research continues, and Krespi et al. combined the actual needs of users, according to the software engineering development process to design the server system. While realizing the access to the server by ordinary PC browser, android application of mobile terminal is developed to realize the mobile terminal [7]. Shi studied and demonstrated the marine environment monitoring system based on Internet of Things technology [8]. Xu et al. designed an intelligent blood glucose monitoring system based on Internet of Things technology and sensor technology [2]. Liu et al. studied the load grade index corresponding to the action, grasped the dynamic change rule of the action according to the movement monitoring index, analyzed the corresponding index of subjective sensation and the method of determining the percentage of exercise intensity, and formulated the calculation formula of the optimal target action and the heart rate index corresponding to the exercise load grade [9]. In the current research, a MEMS-based multiuser motion-monitoring system is proposed. The recognition experiments of seven types of movements show that the proposed deep neural network has a good learning effect on small datasets, reaching 97.61% of the recognition accuracy, and the SVM has also reached over 96% of the recognition accuracy. In the 50 times of operation cycle calculation experiments, the frequency statistics algorithm has reached 100% of the calculation accuracy, and the calculation results of the operation cycle are close to the real value, which proves the validity of the method of cycle calculation.

## 2. Design of Motion-Monitoring System Based on Internet of Things

### 2.1. System Design

A multiuser body movement monitoring system based on MEMS is proposed, and the system consists of sensors, wireless access points, cloud servers, and data receiving terminals. As shown in Figure 1, each sensor node contains a MEMS-based attitude module for collecting action information. Sensors used by multiple users can be connected to a wireless access point through WIFI, and data can be uploaded to the cloud server through the wireless access point. In the cloud server, the machine learning algorithm and wavelet analysis method are used to centrally process the data, and action description information is generated for each user, including action type, action times, and action cycle. The results of motion analysis can be downloaded to any data terminal such as mobile phone or computer through the Internet.

Multiuser action monitoring based on MEMS is a process integrating data acquisition, data transmission, data preprocessing, action recognition, and cycle calculation. The overall algorithm flow is shown in Figure 2. In the research, the nine-axis attitude module based on MPU9250 is used to collect the body motion information, the attitude module can realize the data collection including three-dimensional acceleration, three-dimensional angular velocity and 3D euler angle (angle), at the same time, the initial attitude solution, digital filtering and Kalman filtering are carried out, and the final time-series signal is generated, and the signal is then transmitted through a serial port to the ESP8266 wireless transmission module. The ESP8266 wireless transmission module supports the wifi transmission standard and can upload the action data to the cloud server through the gateway. In order to facilitate debugging, a computer in the local area network is selected as the data processing server, and the action data received by ESP8266 is transmitted to the server through socket for subsequent processing [10, 11]. In the server, the raw data is verified and unpackaged and then stored temporarily as a CSV file, which is still essentially a time-series signal. Next, the motion recognition system reads these files, preprocesses them, and uses pretrained machine learning and deep learning models to identify and classify the movements. Finally, the number statistics and period calculation of the timing signal are carried out based on wavelet and zero-crossing check. After the above steps, a comprehensive description of the categories, times, and periods of an action can be obtained.

The MEMS sensor has its advantages in small volume, low power consumption, and low cost and is widely used in various fields. MEMS-based MEMS human motion information acquisition system uses MEMS accelerometer, MEMS gyroscope, and MEMS magnetometer as the core measurement devices to form its pose measurement unit. The measurement accuracy of the MEMS sensor directly affects the accuracy of the human motion information collection system, so it is necessary to analyze the error of each MEMS sensor used in the human movement information collection system and correct it, which is of great significance for the establishment of the mathematical model of the MEMS sensor.

### 2.2. SVM

In order to realize the motion-monitoring system, MEMS-based inertial sensor is used to collect motion in hardware. In terms of algorithm, SVM is used as one of the classification models with relatively popular and good generalization ability.

Support vector machine (SVM) is one of the most popular supervised learning methods. The proposed action recognition algorithm uses SVM, so the basic theory of SVM is introduced in the following. Before the advent of deep learning, SVM was long regarded as the best performing classification algorithm, especially suitable for application scenarios without any prior knowledge of the relevant field. The main reasons are the following three features of SVM:

1. SVM has good data generalization ability. SVM is a classifier that maximizes the classification interval, the classification hyperplane constructed by SVM ensures the maximum distance to sample points, so it has excellent generalization performance and is not easy to overfit.
2. SVM uses the so-called “kernel method” to map the linearly indivisible data in the low-dimensional plane to the high-dimensional space, making it linearly separable. Therefore, a linear hyperplane generated by SVM in a high-dimensional space is usually not linear in the original space.
3. SVM retains almost all the training samples during the whole process of training and reasoning, which is a nonparametric method. However, only a few training samples play a role in the actual operation, which is called support vector. Therefore, SVM not only has the characteristics of parametric model against overfitting but also has the flexibility of nonparametric model when expressing complex functions.

The use process of SVM can be divided into the training process and reasoning process. The training process is the process of SVM learning rules from the preprepared action samples and delineating the optimal classification hyperplane, and the reasoning process is the process of giving the predicted category according to the data to be tested. Before training the model, the original data of the sensor should be extracted to get the training set. In the training process, the given training set *X* can be expressed as

(1) $$\begin{array}{c} X={\left[x_{1},x_{2},...x_{n}\right]}^{T}, \end{array}$$

where *n* is the number of samples and *x*_*i*_ is the vector representation of the ith training sample.

For SVM, the optimization objective is to find a classification hyperplane with the maximum spacing, and the optimization process can be expressed as

(2) $$\begin{array}{c} \text{min}\frac{1}{2}{\left\|w\right\|}^{2}+C\sum_{i=1}^{n}\zeta_{i}\\ s.t.y\left[\left(wx_{i}\right)+b\right]\geq 1-\varsigma_{i}\left(i=1,2,...,n;\zeta_{i}\geq 0\right), \end{array}$$

where *w* is the normal vector of the classified hyperplane, *b* is the offset, *c* is the penalty coefficient of the support vector machine, *ζ* is the loss term, and *y* is the classification label with A value of +1 or −1. This is a typical convex quadratic programming problem, and its Lagrange coefficient can be obtained by the Lagrange multiplier method, which can be expressed as

(3) $$\begin{array}{c} a=\left[a_{1},a_{2},...a_{n}\right]. \end{array}$$

In essence, the process of SVM optimization in the training phase is the process of finding Lagrange coefficient. In the reasoning stage, the vector representation of the action to be measured and the Lagrange coefficient are substituted into the following formula:

(4) $$\begin{array}{c} g\left(x\right)=\sum_{i=1}^{n}a_{i}y_{i}\left(x_{i},x^{\prime }\right)+b. \end{array}$$

The value of g(x) can be obtained. By comparing the value of g(x) with +1 and −1, the predicted category of the action to be tested can be obtained.

In the framework of support vector machine, Guyon proposed the SVM-RFE feature selection algorithm for sorting features. The core idea of SVM is to establish an optimal.

Hyperplane (*w* · *x*+*b*=0) as decision surfaces and maximizes classification interval (2/‖*w*‖^2^). In dealing with nonlinear and high-dimensional pattern recognition, SVM is linearly separable by mapping kernel function to high-dimensional space. For *l* training sample {(*x*_*i*_, *y*_*i*_), *i*=1,2, ..., *l*} and *x*_*i*_ ∈ *R*^*m*^, *y*_*i*_ ∈ {−1,1}, the objective function satisfying constraint conditions is

(5) $$\begin{array}{c} \left\{\begin{array}{c} \min J=\frac{1}{2}{\left\|w\right\|}^{2}+C\sum_{i=1}^{l}\xi_{i},\\ s.t\left\{\begin{array}{c} y_{i}\left(w\cdot x_{1}+b\right)\geq 1-\xi_{i}\\ \xi_{i}>0 \end{array}\right),i=1,2,...,l. \end{array}\right) \end{array}$$

The decision function of the SVM model is finally obtained by Lagrange duality theorem and quadratic programming:

(6) $$\begin{array}{c} \left\{\begin{array}{c} f\left(x\right)=\mathrm{sgn}\left(w\cdot x+b\right),\\ w=\sum_{i=1}^{l}a_{i}y_{i}x_{i}. \end{array}\right) \end{array}$$

Therefore, in the decision function, the weight *w* is a linear combination of the support vectors whose A is not 0, and the larger the feature weight is, the more discriminant information it contains. In addition, if the ith feature is removed, the influence on the objective function can be calculated by Taylor formula expansion.

(7) $$\begin{array}{c} \Delta J\left(i\right)=\frac{\partial J}{\partial w_{i}}\Delta w_{i}+\frac{\partial^{2}J}{\partial w_{i}^{2}}{\left(\Delta w_{i}\right)}^{2}. \end{array}$$

On the optimal solution of *J*, only the second order is considered, so,

(8) $$\begin{array}{c} \Delta J\left(i\right)\approx {\left(\Delta w_{i}\right)}^{2}. \end{array}$$

When the ith feature is deleted, Δ*w*_*i*_=*w*_*i*_, so, SVM-RFE measures the importance of feature weight and uses w2 as the feature ranking criterion.

## 3. Simulation Experiment

Seven types of body movements were selected for recognition. These movements include four types of dumbbell movements and three types of leg exercises, respectively, dumbbell bending lift, dumbbell side flat lift, dumbbell shoulder push, dumbbell bird, sitting posture leg lift, and standing posture leg lift. These seven kinds of movements are common body exercise movements, with strong representativeness. Among them, there is a high similarity between some movements, such as leg raising by sitting posture and leg raising by standing posture, which poses a certain challenge for the classifier and can fully verify the classification ability of different models. In terms of data, the self-built dataset was used in this study, which was composed of 420 samples in total. A total of six people provided samples for the dataset, including three men and three women, each of whom provided 70 data samples, including 10 for each type of action. When recording data, each participant wore only one attitude acquisition module. For dumbbell action, the posture acquisition module is worn at the wrist. For lower limb movements, the posture acquisition module is worn at the ankle. The weight of the dumbbell used in the dumbbell action is 2.5 kg. In terms of data set allocation, 80% of all samples are used as training set and 20% as the test set. For the deep learning model, 20% of the training set is taken as the verification set.

Figure 3 shows the variation trend of SVM accuracy and loss in training. It can be seen from Figure 3(a) that the training loss and the validation loss continue to decline in the trend until they stop at the 200th training round, during this process, the validation loss is basically consistent with the training loss, in Figure 3(b), the training accuracy and verification accuracy always rise in the trend, and the final difference is not significant, which indicates that the model has learned the law in the data well to a certain extent.

As can be seen from the abovementioned experimental results, SVM achieves the recognition accuracy of more than 96%, higher than the comparison algorithm, while the accuracy of the multilayer perceptron is the lowest among the four models. It can be seen that in 84 test samples, only two dumbbell shoulder pushes were mistakenly classified into dumbbell side lift, which indicates that the SVM model proposed can be well used for action recognition in small datasets. As can be seen from the confusion matrix of SVM, this method is prone to misclassification for the two types of leg movements, which is because the two types of movements are similar, SVM does not perfectly separate the two types of actions based on features from a single sensor. Although SVM does not reach the highest accuracy, it does not have an obvious gap with the deep learning model, so it is more suitable for scenarios with low computing power and also has practical significance.

The purpose of the experiment is to verify the accuracy of counting and cycle calculation. For this experiment, whether the results are objective or not is largely affected by the number of trials. Especially for the action count, the effectiveness of the analysis method can be demonstrated only when the result is still accurate under the condition of sufficient number of times. In this experiment, 50 movements were repeated, which is much higher than the number of times required for a single exercise and can verify the accuracy of the algorithm. In the experimental process, in addition to the use of sensors to record the action, it also uses a stopwatch to time the cycle of each action, as the actual standard.

Table 1 shows the sensitive axes of the seven movements in the dataset obtained according to the abovementioned calculation method. It can be seen that for the movements of the limbs rotating around the joints, the sensitive axis is generally angular velocity, for vertical limb movements such as shoulder push and heel lift, the sensitive axis is acceleration.

Next, the experiment took dumbbell bending as an example, repeated 50 times, and calculated the number of times and period according to the sensitive axis data. Finally, the measured value was compared with the actual value and analyzed. In this experiment, the calculated and actual values of 50 precise cycles are shown in Figure 4. The dotted line marked with the box is the measured value obtained by the calculation method of using the period, the solid line marked with the triangle is the actual value recorded by using the stopwatch, the vertical axis is the period of action in seconds, and the horizontal axis is the number of actions.

Firstly, it can be seen from the length of the curve in the figure that the action count of the algorithm is very accurate, and the statistical result of 50 times is completely consistent with the actual value. Secondly, the overall fitting of the two curves in the figure is good, with an average error of only 0.08s and an average error rate of 4.03%. The maximum error of the calculated results is 0.25s, and the maximum error rate is 13.5%, which occurs only at the end points of the curve. Therefore, the experiment proves that the method of zero-crossing detection and wavelet analysis has a good overall effect and can realize the action count and period calculation more accurately even when the number of actions is more.

As people's attention to sports gradually improve, the concept of healthy life, based on MEMS sports information collection system has extremely important application value, and people can use the system to get more professional sports guidance, in the process of active participation in sports to prevent sports damage, at the same time, the system with big data technology can achieve a more comprehensive sports information analysis function. In this case, the MEMS-based on human movement information collection system adopts modular and miniaturization design, by a variety of measurement units that meet the standards of wearable devices and higher accuracy of attitude estimation algorithm and positioning algorithm, effectively improving the information collection accuracy of the system and applicability and expansion ability in different application scenarios.

## 4. Conclusions

A MEMS-based multiuser motion-monitoring system is proposed to monitor the three important parameters of movement type, movement times, and movement cycle in body movement and to support multiuser simultaneous use. The specific content of the method are as follows: (1) In terms of system design, a motion-monitoring system framework based on the Internet of Things is proposed considering the motion-monitoring scene oriented to intelligent fitness. (2) In the aspect of algorithm, the relevant research of motion pattern recognition and cycle calculation method is carried out. For action pattern recognition, the SVM-based algorithm to adapt to different computing capabilities of the scene is used. (3) In the aspect of system development, the hardware platform including data acquisition bracelet, wireless access point, and PC is developed as well as the software platform integrating data receiving, action recognition, and cycle computing module. The hardware platform and the software platform jointly constitute the experimental platform. Related experiments are carried out based on the developed software and hardware platform. Experiments on 7 kinds of actions show that the proposed deep neural network has a good learning effect on small data sets, the recognition accuracy of the proposed deep neural network reaches 97.61%, and the recognition accuracy of SVM also reaches over 96%. In the 50 times of operation cycle calculation experiments, the frequency statistics algorithm has reached 100% of the calculation accuracy, and the calculation results of the operation cycle are close to the real value, which proves the validity of the method of cycle calculation. In the research process, there are still the following parts to be improved: (1) This system adopts a single sensor to collect limb movement data, which is more convenient in use but can only be used for the movement of a single limb, in the subsequent research, multiple sensors can be installed and the data of multiple sensors can be fused to realize the recognition of complex body movements. (2) Limited by the experimental conditions, the number of training data sources is small; in addition, the cloud server can be replaced by a computer in the lan in the experiment. In subsequent studies, the number of subjects can be increased and the data processing system software can be run using a remote server.

## Figures and Tables

**Figure 1:** Hardware framework of multiuser action monitoring system.

**Figure 2:** Algorithm framework of action monitoring system.

**Figure 3:** (a) Changes in training loss and validation loss. (b) Changes in training accuracy and verification accuracy.

**Figure 4:** Action count and cycle calculation results.

**Table 1:** Sensitive axes for different actions.

Action type	Sensitive axis
Bending	Angular velocity on the *X*-axis
Levelly obeying	Angular velocity on the *X*-axis
Shoulder vertebra	Y-acceleration
The birds	X angular velocity
Seated leg lifts	Z angular velocity
Standing leg lifts	Z angular velocity
Lift heel	Y-acceleration

## Data Availability

The data used to support the findings of this study are available from the corresponding author upon request.
